# lncRNA RHPN1-AS1 Serves as a Sponge for miR-3133 Modulating the Cell Proliferation of Retinoblastoma through JAK2

**DOI:** 10.1155/2020/3502981

**Published:** 2020-12-22

**Authors:** Zhao-Na Li, Ming-Xu Ge, Li-Jun Cao, Zhong-Fang Yuan

**Affiliations:** ^1^Department of Ophthalmology, The Second People's Hospital of Jinan, Jinan, Shandong 250001, China; ^2^Department of Neurosurgery, Shandong Provincial Hospital, Jinan, Shandong 250021, China; ^3^Department of Ophthalmology, Jinan Central Hospital, Cheeloo College of Medicine, Shandong University, Jinan, Shandong 250013, China

## Abstract

**Purpose:**

To investigate the effects of lncRNA RHPN1-AS1 on retinoblastoma (RB) and further explore its underlying molecular mechanisms.

**Methods:**

The expression of RHPN1-AS1, miR-3133, (JAK2), and signal transducer and activator of transcription 3 (STAT3) was detected by qRT-PCR. CCK-8, EDU, and flow cytometry assays were conducted to assess the proliferation activity and apoptosis of RB cells. Double fluorescein and RNA immunoprecipitation assays were performed to detect the interaction between RHPN1-AS1 and miR-3133 or miR-3133 and JAK2. Western blotting was performed to detect the expression of apoptosis-related proteins.

**Results:**

In RB cells, RHPN1-AS1 was upregulated. Silencing RHPN1-AS1 inhibited the activity of RB cells and promoted apoptosis. The expressions of proapoptotic factors (Bax and p53) were increased, while antiapoptotic factors (Bcl-2 and Survivin) were suppressed in siRHPN1-AS1 groups. Furthermore, we predicted and verified that RHPN1-AS1 regulated RB progression by targeting miR-3133/JAK2. In addition, siRHPN1-AS1 also inhibited oncogene STAT3 protein expression.

**Conclusion:**

lncRNA RHPN1-AS1 served as a sponge for miR-3133 to counteract miR-3133-mediated JAK2/STAT3 suppression, indicating that the lncRNA RHPN1-AS1 may be a potential therapeutic target for the treatment of RB.

## 1. Introduction

Retinoblastoma (RB) is a malignant tumor derived from photoreceptor precursor cells that occurs in children, usually under 5 years of age [1]. There are approximately 8000 newly diagnosed retinoblastoma cases worldwide each year [2]. RB has an excellent prognosis where more than 95% of patients survive their disease and approximately 2 thirds of eyes are salvaged [3]. In the developing countries, most patients with retinoblastoma have a poor prognosis, which is usually due to a lack of multidisciplinary care [4]. RB extends along the optic nerve to the brain and is easily transferred [5]. At present, surgery and chemotherapy are still the main antitumor strategies, but chemotherapy has side effects [6]. Therefore, it is urgent to find useful biomarkers and explore new targets for the treatment of RB.

Long noncoding RNAs (lncRNAs) are noncoding RNAs greater than 200 nucleotides in length [7]. Studies have shown that lncRNAs play an important role in many life activities such as dose compensation effect, epigenetic regulation, cell cycle regulation, and cell differentiation regulation [8, 9]. In recent years, lncRNA has become a focus of research, and more importantly, increasing researches have proved that lncRNA can inhibit or promote cancer in different types of cancer [10–12]. Current studies have found that some lncRNAs, which may be involved in tumorigenesis and development, are differentially expressed in tumor tissues and normal tissues [13]. For example, Qiu et al. have demonstrated that lncRNA RHPN1-AS1 is overexpressed in uveal melanoma and non-small-cell lung cancer [14, 15]. In addition, overexpressed RHPN1-AS1 is significantly associated with malignant tumors and poor prognosis. In contrast, downregulation of RHPN1-AS1 inhibits the cell proliferation and metastasis of cancer cells [16]. Although there have been many reports of lncRNA RHPN1-AS1 in tumor development and progression, however, the biological function of lncRNA RHPN1-AS1 in RB cells is rarely explored let alone the underlying molecular mechanisms.

Herein, our results demonstrated an increased expression of RHPN1-AS1 in Y79 and WERI-Rb1, whereas silencing RHPN1-AS1 promoted Y79 and WERI-Rb1 apoptosis. These results suggested that lncRNA RHPN1-AS1 may act as a molecular target of RB.

## 2. Materials and Methods

### 2.1. Cell Culture

Human retinoblastoma (RB) cell lines (Y79 and WERI-Rb1) and human retinal pigment epithelial cell line ARPE-19 were obtained from the American Type Culture Collection (ATCC, Manassas, VA). All cells were cultured in RPMI-1640 medium supplemented with 10% FBS in a humidified environment at 37°C.

### 2.2. Cell Transfection

RHPN1-AS1-siRNA, JAK2-siRNA, small interfering negative control, miR-3133 mimic, miR-NC, and miR-3133 inhibitor were designed and obtained from GenePharma (Shanghai, China). When the confluence rate of cell culture reached 70%, according to the manufacturer's instruction, Lipofectamine 2000 was used to transfect and quantitative real-time PCR (qRT-PCR) was conducted to detect the transfection efficiency.

### 2.3. Quantitative Real-Time PCR

TRIzol reagent was used for the extraction of total RNA, and PrimeScript RT Master Mix Kit was used for reverse transcription. After the sample is prepared, the expression level was detected with SYBR green, and *β*-actin was controlled as an internal parameter followed by the relative fold change analysis by the 2^−*ΔΔ*CT^ method.

### 2.4. Western Blotting Assay

According to the manufacturer's instruction, the proteins were extracted and their concentration was measured. Subsequently, the prepared protein was separated by polyacrylamide-SDS gels and electroblotted onto nitrocellulose membranes. After 2 h of blocking, the membrane incubated overnight against primary antibodies: p53, Bax, Bcl-2, Survivin, JAK2, STAT3, and *β*-actin followed by the secondary antibody for 30 min at 37°C. The intensity of protein expression was detected by ECL chemiluminescence.

### 2.5. Cell Counting Kit-8 (CCK-8) Assay

The proliferation activity of Y79, WERI-Rb1, and ARPE-19 was detected by the CCK-8 assay (Beyotime, Beijing, China). In short, the cells in the logarithmic phase were inoculated on a 96-well plate and treated accordingly. Then, after washing with phosphate buffer solution (PBS) for three times, the indicated cells were incubated with CCK-8 for 2 h at 37°C. Finally, the absorbance was measured at 450 nm.

### 2.6. EDU Assay

The proliferation ability of Y79 and WERI-Rb1 was evaluated by the EDU assay. Briefly, after transfection, Y79 and WERI-Rb1 were seeded in 96-well plates for 48 h. Following, Y79 and WERI-Rb1 were incubated with 10 *μ*M EDU for 2 h at 37°C degrees ambient temperature, followed by washing with PBS. EDU-positive cells were detected by Apollo staining and DAPI staining, and the percentage of positive cells was defined as the proliferation rate.

### 2.7. Flow Cytometry

Transfected Y79 and WERI-Rb1 cells were incubated with Annexin V in the dark for 20 minutes. Subsequently, 10 *μ*L propidium iodide (PI) was also added to the cell suspension, and the apoptosis rate of the cells was measured by a flow cytometer (BD Biosciences, CA, USA).

### 2.8. Bioinformatics

DIANA tools (http://carolina.imis.athena-innovation.gr/diana_tools/web/index.php) were used to predict the interaction of lncRNA RHPN1-AS1 and miR-3133. TargetScan (http://www.targetscan.org/vert_72/) was used to predict the interaction of miR-3133 and JAK2.

### 2.9. Luciferase Reporter Assay

Wt-RHPN1-AS1, mut-RHPN1-AS1, Wt-JAK2, and mut-JAK2 were inserted into pmirGLO reporter vectors (Promega, Madison, WI, USA), respectively. Y79 and WERI-Rb1 were plated onto 24-well plates and cotransfected with vectors of the above constructed and miR-3133 mimics or mimic-NC. Luciferase activities were determined with the Dual-Luciferase Reporter System (Promega, Madison, WI, USA).

### 2.10. RNA Immunoprecipitation (RIP) Assay

RIP was performed by using the Magna RIP RNA-Binding Protein Immunoprecipitation Kit (Millipore, Bedford, MA). Briefly, cultured Y79 and WERI-Rb1 cells were collected and resuspended in RIP lysis buffer (Solarbio), and the cell extracts were incubated with RIP buffer containing magnetic beads conjugated with human anti-Ago2 antibody (Millipore) or control IgG (Merck Millipore) at room temperature overnight. Subsequently, the magnetic beads were incubated with proteinase K after washing three times. Total RNA was subsequently isolated from the extracts using TRIzol. The relative enrichments of lncRNA RHPN1-AS1 and miR-3133 were determined by qRT-PCR analysis.

### 2.11. Statistical Analysis

All the data were analyzed by SPSS 19.0 (SPSS, Chicago, IL, USA) and presented as mean ± standard deviation. Student's *t*-test or one-way ANOVA followed by Dunnett's multiple comparison was applied to assess the differences between groups. A *P* < 0.05 was considered statistically significant.

## 3. Results

### 3.1. Silencing of RHPN1-AS1 Inhibited the Proliferation of RB Cell Lines and Promoted Their Apoptosis

As indicated in Figure 1(a), the mRNA expression of RHPN1-AS1 in Y79 and WERI-Rb1 was obviously higher than that in the ARPE-19 cells. To further investigate the role of lncRNA RHPN1-AS1 on RB, Y79 and WERI-Rb1 cells were then transfected with siRHPN1-AS1 or siNC and we found that there was a decreased expression of RHPN1-AS1 in the siRHPN1-AS1 group when compared with the siNC group (Figure 1(b)). Next, we performed the CCK-8 assay, EDU assay, and flow cytometry assay to detect the effects of silencing RHPN1-AS1 on RB cell line proliferation and apoptosis. The CCK-8 and EDU results indicated that silencing of RHPN1-AS1 inhibited the proliferation ability of Y79 and WERI-Rb1 (Figures 1(c) and 1(d)), while the flow cytometry results showed that silencing RHPN1-AS1 remarkably induced the apoptosis of RB cells (*P* < 0.001; Figure 1(f)). p53, Bax, Bcl-2, and Survivin are all apoptosis-related genes; therefore, to further detect the effect of the role of RHPN1-AS1 in the progression of RB, western blotting was conducted. As expected, silencing of RHPN1-AS1 can promote the expression of proapoptotic factors Bax and p53 and inhibit the protein expression of antiapoptotic factors Bcl-2 and Survivin (Figure 1(e)).

### 3.2. miR-3133 Is a Target of RHPN1-AS1 in RB Cells

As predicted by DIANA tools, miR-3133 may be the target microRNA. To confirm this conjecture, two types of luciferase reporter gene vectors (RHPN1-AS1-wt and RHPN1-AS1-mut) were conducted in this study to investigate whether lncRNA RHPN1-AS1 serves as a sponge for miR-3133 by direct binding (Figure 2(a)). As shown in Figure 2(b), after being transfected with RHPN1-AS1-wt, miR-3133 mimic significantly inhibited relative luciferase activity. However, when we mutate out this predicted binding site, overexpression of miR-3133 did not change the activity of luciferase. The RIP assay showed that the Ago2 antibody was able to pull down both endogenous RHPN1-AS1 and miR-3133 (Figure 2(c)), further validating their binding potential. To further verify the interaction between RHPN1-AS1 and miR-3133, Y79 and WERI-Rb1 were transfected with siRHPN1-AS1, miR-3133 inhibitor, or the corresponding negative control. Compared with siNC, transfection of siRHPN1-AS1 could promote the expression of miR-3133. When added with miR-3133 inhibitor, the miR-3133 expression was remarkably decreased in comparison to the siRHPN1-AS1 group (Figure 2(d)). In Figure 2(e), the mRNA expression of miR-3133 in Y79 and WERI-Rb1 was obviously lower than that in the ARPE-19 cells, which is consistent with the previous expression result of RHPN1-AS1 inhibiting miR-3133 expression.

### 3.3. miR-3133 Inhibitor Eliminated the Role of siRHPN1-AS1 in RB Cells

We have proved that lncRNA RHPN1-AS1 is a sponge for miR-3133 to negatively regulate its expression. Next, to further demonstrate the role of the interaction between the two in RB progression, we added an inhibitor of miR-3133. CCK-8 and EDU results showed that the proliferation of cells transfected with siRHPN1-AS1 was restored after the addition of miR-3133 inhibitor (Figures 3(a) and 3(b)). Similarly, the flow cytometry assay confirmed that miR-3133 inhibitor inhibited the apoptosis of Y79 and WERI-Rb1 after being transfected with siRHPN1-AS1 (Figure 3(d)). Western blotting results also showed that after adding miR-3133 inhibitor, the expression of p53 and Bax was also significantly reduced, while the expression of Bcl-2 and Survivin was significantly increased (Figure 3(c)).

### 3.4. JAK2 Is a Target of miR-3133 in RB Cells

As predicted by TargetScan, JAK2 was the downstream target mRNA of miR-3133 (Figure 4(a)). Therefore, we conducted JAK2-wt and JAK2-mut luciferase reporter plasmids to transfect miR-3133 mimic or mimic-NC to Y79 and WERI-Rb1 cells for luciferase assay. In Figure 4(b), after being transfected with JAK2-wt, miR-3133 mimic significantly inhibited relative luciferase activity. However, after mutating the predicted binding site, miR-3133 mimic had no effect on the luciferase activity. Besides, we detected the mRNA expression changes of JAK2 by qRT-PCR. The qRT-PCR results showed that miR-3133 overexpression significantly reduced the mRNA expression of JAK2 in Y79 and WERI-Rb1. However, when the miR-3133 inhibitor was added, significant upregulation of JAK2 mRNA expression was observed in comparison to miR-3133 mimic (Figure 4(c)).

### 3.5. lncRNA RHPN1-AS1 Regulated RB Cells by Targeting miR-3133/JAK2

To further explore the underlying molecular mechanism of lncRNA RHPN1-AS1 regulating RB, qRT-PCR and western blotting were conducted. In Figure 5(a), silencing RHPN1-AS1 significantly downregulated JAK2 expression in Y79 and WERI-Rb1, while adding miR-3133 inhibitor could counteract the inhibitory effect of siRHPN1-AS1 on JAK2. Moreover, we also tested the expression level of another oncogene, STAT3, after corresponding treatment. As expected, the mRNA expression of STAT3 was remarkably decreased after transfection with siRHPN1-AS1. Conversely, the addition of miR-3133 inhibitor restored the mRNA expression of STAT3 (Figure 5(a)). Similarly, the western blotting assay confirmed that siRHPN1-AS1 inhibited the protein expression of JAK2 and STAT3 (Figure 5(b)).

### 3.6. Silencing of JAK2 Inhibited the Proliferation of RB Cell Lines and Promoted Their Apoptosis

As indicated in Figure 6(a), the protein expression of JAK2 in Y79 and WERI-Rb1 was markedly higher than that in the ARPE-19 cells. To further investigate the role of JAK2 on RB, Y79 and WERI-Rb1 cells were then transfected with siJAK2 or siNC and we found that there was a decreased expression of JAK2 in the siJAK2 group when compared with the siNC group (Figure 6(b)). The CCK-8 and EDU results indicated that silencing of JAK2 inhibited the proliferation ability of Y79 and WERI-Rb1 (Figures 6(c) and 6(d)), while the flow cytometry results showed that silencing JAK2 remarkably induced the apoptosis of RB cells (*P* < 0.01; Figure 6(e)).

### 3.7. siJAK2 Abrogated the Role of miR-3133 Inhibitor in RB Cells

CCK-8 and EDU results showed that the proliferation of cells transfected with *miR-3133 inhibitor* was restored after the addition of siJAK2 (Figures 7(a) and 7(b)). Similarly, the flow cytometry assay confirmed that siJAK2 inhibited the apoptosis of Y79 and WERI-Rb1 after being transfected with *miR-3133 inhibitor* (Figure 7(c)).

## 4. Discussion

In recent years, lncRNAs regulate various cellular processes, such as cell proliferation, metastasis, differentiation, and metabolism, leading to the progression of many diseases including malignant tumors [14]. In the presented study, we showed an upregulation of lncRNA RHPN1-AS1 in Rb cell lines when compared with ARPE-19 cells and silencing of lncRNA RHPN1-AS1 promoted apoptosis of Y79 and WERI-Rb1 cells. Mechanistically, we proved lncRNA RHPN1-AS1 to counteract miR-3133-mediated JAK2 suppression by acting as a sponge for miR-3133.

RHPN1-AS1 gene is located on the chromosome 8q24.3 and is derived from the promoter region of the RHPN1 gene. lncRNA RHPN1-AS1 is a key regulator of disease progression in many cancer types, but its biological function has not been widely reported [15]. Early studies have reported that RHPN1-AS1 is highly expressed in uveal melanoma cancer tissues and cell lines, and RHPN1-AS1, an oncogene, promotes the progression of uveal melanoma [16]. In addition, RHPN1-AS1 is also found highly expressed in human breast cancer tissues and MCF-7 cell lines and further mechanism studies have shown that RHPN1-AS1 promotes tumorigenesis by modulating the expression of p53 [17]. Importantly, bioinformatics analysis has shown a significant correlation between RHPN1-AS1 and the onset, development, and metastasis of cancer [18]. Consistent with the above finding, there was an increased expression of RHPN1-AS1 in RB cells compared to ARPE-19 cells in our study. More importantly, silencing of RHPN1-AS1 greatly inhibited the proliferation and promoted apoptosis of Y79 and WERI-Rb1 cells. The apoptosis of cells can be regulated by specific proteins, thereby regulating tumorigenesis and progression. Among these specific apoptosis-related proteins, Bax can promote the apoptosis of cancer cells, while Bcl-2 can interact with Bax to regulate the occurrence of apoptosis [19]. p53 is also an important gene involved in apoptosis, which can promote apoptosis by upregulating Bax expression and downregulating Bcl-2 expression [20]. Survivin is a newly discovered protein belonging to the apoptosis-inhibiting protein family, and it is found the strongest apoptosis-inhibiting factor found so far. In our study, we found that p53 and Bax were upregulated, while Bcl-2 and Survivin were downregulated after RHPN1-AS1 was silenced. Collectively, the above finding indicates that lncRNA RHPN1-AS1 was involved in the behavior of RB cells.

It has been reported that lncRNA can regulate the occurrence and development of tumors by targeting microRNAs (miRNAs) [21]. Usually, lncRNA acts as a miRNA sponge to offset miRNA-mediated inhibition of its downstream targets or signaling pathways [22], thereby exerting its biological function. Previously, miR-3133 has been reported to be downregulated in clear cell renal cell carcinoma (ccRCC) and play an inhibitory role in the aggressive progression of ccRCC [23]. In this study, we used DIANA tools to predict miR-3133 was the downstream target of RHPN1-AS1.

The direct binding between miR-3133 and RHPN1-AS1 was confirmed by double fluorescein and RIP assays, and from the results of this experiment, we found the expression of miR-3133 and RHPN1-AS1 in Y79 and WERI-Rb1 negative correlation. Furthermore, we detected the proliferation, apoptosis, and apoptosis-related protein expression of RB cell, which were transfected with siRHPN1-AS1 or miR-3133 inhibitor. As the study showed, silencing of RHPN1-AS1 inhibited RB proliferation, while miR-3133 inhibition, on the contrary, partially counteracted the effects of RHPN1-AS1 knockout. The above results indicate that lncRNA RHPN1-AS1 acted as a sponge to regulate the proliferation of RB cells.

miRNAs are a class of short noncoding RNA molecules that negatively regulate gene expression, thereby degrading their targeted mRNAs and inhibiting their transplantation [23, 24]. JAK2 is a member of the Janus family of tyrosine kinases, which encodes a protein that is a nonreceptor tyrosine kinase and is involved in many important biological processes, such as cell proliferation, differentiation, apoptosis, and immune regulation [25]. In our study, we used TargetScan to predict that JAK2 was the target of miR-3133, and we confirmed this prediction. Further, we proved that JAK2 has a negative regulatory relationship with miR-3133. When miR-3133 was overexpressed in Y79 and WERI-Rb1, the mRNA expression of JAK2 was reduced significantly. On the contrary, when the miR-3133 inhibitor was added, the expression of JAK2 was significantly upregulated. To further verify the above prediction, we transfected RB cell lines with siRHPN1-AS1 or miR-3133 inhibitor. We found that RHPN1-AS1 knockdown inhibited the expression of JAK2. More interestingly, the addition of miR-3133 inhibitor restored the expression of JAK2 to a certain extent. Signal transducer and activator of transcription 3 (STAT3) is a member of the seven protein family [26], and it could regulate the transcription of a number of genes associated with oncogenic behavior, such as proliferation, apoptosis, invasion, and metastasis [27] and can be activated by upstream JAK2 (Janus Kinase 2) [28, 29]. Therefore, we also detected changes in the expression of STAT3. As expected, knockout RHPN1-AS1 also inhibited the expression of STAT3 in Y79 and WERI-Rb1, which was consistent with the expression pattern of JAK2. Collectively, our results indicated that the role of lncRNA RHPN1-AS1 in RB progression may be related to the expression of miR-3133/JAK2.

## 5. Conclusion

In our study, RHPN1-AS1 was upregulated in RB cell lines. Further, lncRNA RHPN1-AS1 was negatively correlated with miR-3133 and positively correlated with JAK2/STAT3. Taken together, RHPN1-AS1/miR-3133/JAK2 may be a promising molecular target for RB.

## Figures and Tables

**Figure 1:** Silencing of RHPN1-AS1 inhibited the proliferation of RB cell lines and promoted their apoptosis. (a) lncRNA RHPN1-AS1 was upregulated in RB cell lines; ^∗∗^*P* < 0.01, compared with APRE-19; (b) lncRNA RHPN1-AS1 expression was detected after transfection with siRHPN1-AS1 or siNC in Y79 and WERI-Rb1; ^∗∗^*P* < 0.01, compared with siNC; (c) the proliferation activity of Y79 and WERI-Rb1 was detected by CCK-8; ^∗^*P* < 0.05 and ^∗∗^*P* < 0.01, indicated compared with 0 h; (d) cell proliferation of Y79 and WERI-Rb1 cells was identified by the EDU assay; (e) western blotting was used to detect the expression of apoptosis-related proteins; ^∗∗^*P* < 0.01, compared with siNC; (f) after transfection with siRHPN1-AS1 or siNC, the apoptosis of Y79 and WERI-Rb1 cells was detected by flow cytometry; ^∗∗^*P* < 0.01, compared with siNC.

**Figure 2:** miR-3133 is a target of RHPN1-AS1 in RB cells. (a) There is a complementary binding region between miR-3133 and RHPN1-AS1 (DIANA tools); (b) wt-RHPN1-AS1 or mut-RHPN1-AS1 was cotransfected with miR-3133 mimics; then, the relative luciferase activity was evaluated by the luciferase reporter assay; ^∗∗^*P* < 0.01, compared with wt-RHPN1-AS1; (c) the RIP assay was performed with cell extracts of Y79 and WERI-Rb1. Ago2 and IgG antibodies were used for immunoprecipitation, and qRT-PCR was performed to detect the relative RNA level of RHPN1-AS1 or miR-3133. (d) miR-3133 mRNA expression in Y79 and WERI-Rb1 was examined by qRT-PCR; ^∗∗^*P* < 0.01, compared with siNC+inhibitor NC; (e) compared with APRE-19, miR-3133 was downregulated in RB cell lines.

**Figure 3:** miR-3133 inhibitor eliminated the role of siRHPN1-AS1 in RB cell. (a) The cell proliferation of Y79 and WERI-Rb1 was detected by CCK-8 after transfection with siRHPN1-AS1 or miR-3133 inhibitor; ^∗^*P* < 0.05, compared with 0 h; (b) the EDU assay was used to detect the cell proliferation of Y79 and WERI-Rb1 cells; ^∗∗^*P* < 0.01, compared with siNC+inhibitor NC; (c) protein expression of p53, Bax, Bcl-2, and Survivin was detected after transfection with siRHPN1-AS1 or miR-3133 inhibitor; (d) RB cells (Y79 and WERI-Rb-1) were transfected with siRHPN1-AS1 or miR-3133 inhibitor, and apoptosis was detected by flow cytometry; ^∗^*P* < 0.05 and ^∗∗^*P* < 0.01, indicated compared with siNC+inhibitor NC.

**Figure 4:** JAK2 is a target of miR-3133 in RB cells. (a) A binding site between miR-3133 and JAK2 was predicted by the TargetScan; (b) after cotransfection with miR-3133 mimics and wt-JAK2 or mut-JAK2, the luciferase activity was detected by the double fluorescein assay; ^∗∗^*P* < 0.01, compared with wt-JAK2; (c) JAK2 mRNA expression in Y79 and WERI-Rb1 was examined by qRT-PCR; ^∗∗^*P* < 0.01, indicated compared with mimics NC; ^##^*P* < 0.01, indicated compared with inhibitor NC.

**Figure 5:** lncRNA RHPN1-AS1 regulated RB cells by targeting miR-3133/JAK2. (a) The mRNA expression of JAK2 and STAT3 was detected after transfection with siRHPN1-AS1 or miR-3133 inhibitor; ^∗^*P* < 0.05 and ^∗∗^*P* < 0.01, compared with siNC+inhibitor NC; (b) the protein expression of JAK2 and STAT3 was detected after transfection with siRHPN1-AS1 or miR-3133 inhibitor.

**Figure 6:** Silencing of JAK2 inhibited the proliferation of RB cell lines and promoted their apoptosis. (a) lncRNA RHPN1-AS1 was upregulated in RB cell lines; ^∗∗^*P* < 0.01, compared with APRE-19; (b) the protein expression JAK2 was detected after transfection with siJAK2 or siNC in Y79 and WERI-Rb1; ^∗∗^*P* < 0.01, compared with siNC; (c) the proliferation activity of Y79 and WERI-Rb1 was detected by CCK-8; ^∗^*P* < 0.05 and ^∗∗^*P* < 0.01, indicated compared with 0 h; (d) cell proliferation of Y79 and WERI-Rb1 cells was identified by the EDU assay; (e) after transfection with siJAK2 or siNC, the apoptosis of Y79 and WERI-Rb1 cells was detected by flow cytometry; ^∗∗^*P* < 0.01, compared with siNC.

**Figure 7:** siJAK2 abrogated the role of miR-3133 inhibitor in RB cell. (a) The cell proliferation of Y79 and WERI-Rb1 was detected by CCK-8 after transfection with siJAK2 or miR-3133 inhibitor; ^∗^*P* < 0.05, compared with 0 h; (b) the EDU assay was used to detect the cell proliferation of Y79 and WERI-Rb1 cells; ^∗∗^*P* < 0.01, compared with siNC+inhibitor NC; (c) RB cells (Y79 and WERI-Rb-1) were transfected with siJAK2 or miR-3133 inhibitor, and apoptosis was detected by flow cytometry; ^∗^*P* < 0.05 and ^∗∗^*P* < 0.01, indicated compared with siNC+inhibitor NC.

## Data Availability

The datasets used and analyzed during the current study are available from the corresponding author on reasonable request.
